The article "Potentiation of the Activity of Antibiotics against ATCC and MDR Bacterial Strains with (+)-α-Pinene and (-)-Borneol" was published in 2022. Journal: Biomed Res Int.

# Potentiation of the Activity of Antibiotics against ATCC and MDR Bacterial Strains with (+)-*α*-Pinene and (-)-Borneol

**DOI:** 10.1155/2022/8217380

**Published:** 2022-05-25

**Authors:** Nadghia F. Leite-Sampaio, Cicera N. F. L. Gondim, Rachel A. A. Martins, Abolghasem Siyadatpanah, Roghayeh Norouzi, Bonglee Kim, Celestina E. Sobral-Souza, Gonçalo E. C. Gondim, Jaime Ribeiro-Filho, Henrique D. M. Coutinho

**Affiliations:** ^1^Regional University of Cariri-URCA, Crato, Brazil; ^2^Ferdows School of Paramedical and Health, Birjand University of Medical Sciences, Birjand, Iran; ^3^Department of Pathobiology, Faculty of Veterinary Medicine, University of Tabriz, Tabriz, Iran; ^4^Department of Pathology, College of Korean Medicine, Kyung Hee University, Seoul 02447, Republic of Korea; ^5^Vale do Salgado University Center, Icó, Brazil; ^6^Institute of Technological Education Center/Cariri, Juazeiro do Norte, Brazil; ^7^Gonçalo Moniz Institute (IGM), Oswaldo Cruz Foundation (Fiocruz), Salvador, Bahia, Brazil

## Abstract

The increasing rates of antimicrobial resistance have demanded the development of new drugs as conventional antibiotics have become significantly less effective. Evidence has identified a variety of phytocompounds with the potential to be used in the combat of infections caused by multidrug-resistant (MDR) bacteria. Considering the verification that terpenes are promising antibacterial compounds, the present research aimed to evaluate the antibacterial and antibiotic-modulating activity of (+)-*α*-pinene and (-)-borneol against MDR bacterial strains. The broth microdilution method was used to determine the minimum inhibitory concentration (MIC) of the compounds and antibiotics and further evaluate the intrinsic and associated antibiotic activity. These analyses revealed that (+)-*α*-pinene showed significant antibacterial activity only against *E. coli* (MIC = 512 *μ*g.mL^−1^), while no significant inhibition of *S. aureus* and *P. aeruginosa* growth was observed (MIC ≥ 1024 *μ*g mL^−1^). However, when combined with antibiotics, this compound induced a significant improvement in the activity of conventional antibiotics, as observed for ciprofloxacin, amikacin, and gentamicin against *Staphylococcus aureus*, as well as for amikacin and gentamicin against *Escherichia coli*, and amikacin against *Pseudomonas aeruginosa*. On the other hand, (-)-borneol was found to inhibit the growth of *E. coli* and enhance the antibiotic activity of ciprofloxacin and gentamicin against *S. aureus*. The present findings indicate that (+)-*α*-pinene and (-)-borneol are phytocompounds with the potential to be used in the combat of antibacterial resistance.

## 1. Introduction

In the last decades, the treatment of infections has been threatened by the emergence and spread of an increasing variety of pathogens developing resistance mechanisms against antimicrobial drugs. Antimicrobial resistance occurs when microorganisms such as bacteria, viruses, fungi, and parasites present modifications to evade the action of antimicrobial drugs, resulting in increased rates of transmission, morbidity, and mortality [1].

Consistent evidence has indicated that the antibiotic resistance process has been accelerated in recent years due to the inadequate and uncontrolled use of these drugs, which represents an issue of significant concern for future generations [2].

In order to reduce the irrational use of antimicrobials, the Brazilian Health Regulatory Agency (ANVISA) has published a resolution [3] to regulate and control the use of antimicrobials drugs so that, either alone or in association, they should be sold exclusively under prescription.

In response to the bacterial resistance threat, researchers have made significant efforts to isolate and identify new compounds with antibacterial properties [4], as conventional antibiotics have become significantly less effective [5]. In this context, the development of studies using plant-derived natural products has been pointed as a promising strategy to accelerate and cheapen the production of novel antibacterial compounds [6].

In fact, the use of medicinal plants for therapeutic purposes is an ancient practice. Currently, it is well-established that the therapeutic properties of medicinal species are due to the presence of secondary metabolites [7] which, besides playing critical physiological roles, can interfere with pharmacological targets in human beings and many other species. Therefore, medicinal plants are relevant sources of new molecules with the potential to be used in drug development [8, 9].

However, the development of new antibiotics is limited by the high cost of the process and the restrictions on profits compared to other drugs. In addition, the clinical benefits of antibiotics can decrease over time, so their use needs to be restricted to prevent antibacterial resistance [10].

Terpenes are a class of lipophilic hydrocarbon compounds composed of isoprene units. Such physicochemical characteristic favors their interaction with the lipid bilayer of cell membranes. Consequently, terpenoids can induce significant changes in the structure of membrane components in different microorganisms [11–13].

Pinene (C_10_H_16_) is a bicyclic, double-bonded terpenoid hydrocarbon compound [14]. The compound *α*-pinene is found in nature in essential oils (EO) approximately 40 different essential oils. It is among the best-known representatives of an extensive family of monoterpenes. This compound has two enantiomers (+) and (-), which are commercially available and have proven pharmacological activities, among which their antimicrobial properties stand out [15, 16]. Additionally, these isomers present a number of applications, especially in the composition of flavors and fragrances [17] and in the composition of medicines for the treatment of renal and hepatic diseases [18]. Importantly, it has been postulated that the antibacterial properties of *α*- and *β*-pinene are due to their toxic effects on the cell membrane [19].

Borneol is a monoterpene identified in the essential oils of several medicinal plants. It is classified as a bicyclic monoterpenoid alcohol that exists as the D and L enantiomers. This compound has been used in the treatment of gastrointestinal diseases in traditional medicine in China and India [9]. A large number of borneol derivatives have been both designed and synthesized, demonstrating significant activity against *Streptococcus sanguinis*, *Staphylococcus aureus*, *Escherichia coli*, *Pseudomonas aeruginosa*, and *Candida albicans*. Among them, the bornyl 3′,4′-dimethoxybenzoate derivative stood out for its strong activity against several pathogens [20].

Recent research identified a number of pharmacological activities for borneol including neuroprotective [21], analgesic [22, 23], muscle relaxing [24], anti-inflammatory [25], antitumor [26], antiasthmatic [27], and anxiolytic [28]. In addition, due to its antiadhesive antimicrobial properties, borneol has potential applications in multifunctional textiles and healthcare [29].

Consistent evidence has indicated that the effectiveness of combined drugs against microorganisms can be greater than that of isolated antibiotics, which has long been observed from studies analyzing the synergism between natural products and conventional antibiotics [30].

Therefore, considering the verification that terpenes are promising antibacterial compounds, the present research aimed to evaluate the antibacterial and antibiotic-modulating activity of (+)-*α*-pinene and (-)-borneol against MDR bacterial strains.

## 2. Materials and Methods

### 2.1. Bacterial Cultures

The standard bacteria used in the tests were obtained from the American Type Culture Collection, clinical isolates were obtained from the University Hospital of the Federal University of Paraíba, and both were stored under refrigeration (8°C) in slanted test tubes containing heart infusion agar (Heart Infusion Agar-HIA, Difco, USA). The standard bacterial strains *Escherichia coli* ATCC 2592, *Staphylococcus aureus* ATCC 25923, *Pseudomonas aeruginosa* ATCC 9027, and multiresistant isolates of *E. coli* 06, *S. aureus* 10, and *P. aeruginosa* 24 were used in the antibacterial tests. All experimental protocols were carried out at the Laboratory of Microbiology and Molecular Biology (LMMB) of the Regional University of Cariri (URCA). Antibiotic susceptibility testing (Table 1) was performed by Kirby-Bauer's disk diffusion method on Muller-Hinton agar (Hi Media, Mumbai, India) in accordance with the standards of the Clinical Laboratory Standards Institute (CLSI) [31].

### 2.2. Drugs and Reagents

The compounds (+)-*α*-pinene and (-)-borneol were weighed and 10 mg of each substance was diluted in 1 mL of dimethyl sulfoxide (DMSO, purity = 99.9%) and sterile distilled water until reaching a concentration of 1,024 *μ*g/mL. Resazurin, sodium salt (Sigma-Aldrich, St. Louis, MO, USA) was used as a colorimetric indicator of bacterial growth through the oxidation-reduction method [32, 33].

The test substances were prepared as previously described in the literature [34, 35]. The antibiotics, trimethoprim*/*sulfamethoxazole, metronidazole, ciprofloxacin, clindamycin, amikacin, and gentamicin, were dissolved and diluted in sterile water to 1,024 *μ*g/mL.

### 2.3. Strains

Bacterial culture samples were seeded in Petri dishes containing solid heart infusion agar (HIA) medium and stored at 37°C for growth for 24 h. Then, an aliquot of the microbial culture was removed with an inoculation loop and transferred to test tubes containing sterile saline solution (0.9%). The turbidity of the inoculum was compared to the McFarland scale corresponding to 1 × 10^8^ CFU. This test was carried out in triplicate.

### 2.4. Determination of Minimum Inhibitory Concentration (MIC)

The minimum inhibitory concentration (MIC) was defined as the lowest concentration capable of preventing bacterial growth in the microdilution plate wells as detected macroscopically [31]. The MIC was determined using standard nonresistant bacterial strains. To this end, each strain was cultured in three Petri dishes containing HIA. After 24 h, an aliquot of each plate was collected to obtain an inoculum with a final concentration of 10^5^ CFU. Test tubes were filled with 1350 *μ*L of 10% brain heart infusion (BHI) + 150 *μ*L of inoculum. Then, 100 *μ*L of this solution was distributed in each well of 96-well plates. Then, 100 *μ*L of each monoterpene was added to the first well, and a serial dilution was performed in each column of the plate to achieve concentrations ranging from 512 *μ*g/ml to 0.5 *μ*g/ml. The plates were then placed in an incubator for 24 h at 37°C, followed by the addition of 20 *μ*l of resazurin to each well. After 1 h, the reading was carried out by ocular observation of the solution color, so that a change from blue to red or purple was used as an indication of bacterial growth. Of note, according to Houghton et al. [36], a natural product with an effective concentration higher than 1 mg/mL cannot be considered clinically relevant due to the impossibility of achieving adequate plasma concentrations.

### 2.5. Modulation Antibiotic Activity by Direct Contact

The method proposed by Coutinho et al. [37] was used in the analysis of antibiotic activity modulation against MDR isolates. Briefly, the bacterial inoculum was prepared in BHI as described above, and the compounds were added at a subinhibitory concentration (equivalent to its MIC÷8). The wells in a 96-well plate were filled with 100 *μ*L of this solution, followed by the addition of 100 *μ*L of each antibiotic at concentrations ranging from 512 to 0.5 *μ*g/mL. The MIC of each drug in the presence or absence of the natural product was determined, and the occurrence of synergism was interpreted as increased antibiotic activity. Experimental controls and readings were performed as previously described.

### 2.6. Statistical Analysis

The data were analyzed through the statistical program GraphPad Prism version 7.0. The analysis was performed by two-way ANOVA, using the geometric average of the triplicates as the central data and the standard deviation of the average. A Bonferroni post hoc test was then performed, and a *p* < 0.05 was considered significant.

## 3. Results

As shown in Table 2, both (+)-*α*-pinene and (-)-borneol presented a MIC of 512 *μ*g/mL against the ATCC strain of *E. coli*, while MICs ≥ 1024 *μg*/mL were obtained against *S. aureus* and *P. aeruginosa*. Therefore, both compounds were found to present significant antibacterial effects only against *E. coli*.

To evaluate the potentiation of antibiotic activity, we investigated the ability of the natural products to reduce the antibiotic MIC.  Figure 1 shows that the MIC of ciprofloxacin against *S. aureus* was reduced from 101.5 *μ*g/mL to 80.6 *μ*g/mL when associated with (+)-*α*-pinene. The results were even more expressive with the drugs amikacin and gentamicin whose MIC was reduced by 90% and 92%, respectively, against the same strain. On the other hand, the association of (+)-*α*-pinene with the trimethoprim/sulfamethoxazole, metronidazole, and clindamycin had no significant impact on their MIC, indicating an absence of antibiotic activity modulation.

The analysis of antibiotic-enhancing activity of (-)-borneol in *S. aureus* cultures (Figure 2) demonstrated that its association with ciprofloxacin caused a reduction of 37% in the antibiotic MIC. In addition, the association with gentamicin, reduced the antibiotic MIC by 75%, changing from 32 *μ*g/mL to 8 *μ*g/mL, indicating potentiated antibiotic activity.

The analysis of antibiotic resistance modulation by (+)-*α*-pinene against *E. coli* is shown in Figure 3. Among the antibiotics, only amikacin and gentamicin had their MIC changed by the compound. While the MIC of amikacin was reduced from 50.8 *μ*g/mL to 40.3 *μ*g/mL, the MIC of gentamicin was reduced from 20.1 *μ*g/mL to 16 *μ*g/mL.

On the other hand, under the same conditions described above, an antagonistic activity was observed from the combination of (-)-borneol with trimethoprim/sulfamethoxazole against *E. coli*, since the antibiotic MIC increased from 512 *μ*g/mL to ≥1024 *μ*g/mL (Figure 4). However, no significant modulation of antibiotic activity was observed from the association of (-)-borneol with the other drugs.

*P. aeruginosa* was found to present significant resistance to antibiotics, whose MIC was poorly affected by the association with (+)-*α*-pinene. Nevertheless, it is worth mentioning that this monoterpene caused a reduction of 37% in the MIC of amikacin in comparison with the control (Figure 5).

Under the same conditions described above, (-)-borneol failed to modulate the activity of all antibiotics against *P. aeruginosa*, as no significant MIC change was observed (Figure 6).

Discussion

The use of these natural compounds in the treatment of infections is considered a traditional alternative to the use of synthetic drugs [33]. Studies have demonstrated that monoterpenes can improve the activity of antimicrobial drugs, increasing their effectiveness against resistant pathogens, which can accelerate the healing, as well as hinder the microbial adaptability. Resistance to aminoglycosides and other antibacterial drugs has been a major threat to public health. Aminoglycosides inhibit protein synthesis by altering the conformation of the bacterial ribosome [34, 38] presenting enzymatic inactivation and efflux pump expression as major resistance mechanisms [37].

A significant body of research has demonstrated that antibiotic resistance can be reversed using natural products such as extracts, fractions, essential oils, and isolated phytocompounds, as well as their synthetic and semisynthetic derivatives [33, 34, 37, 38]. While the molecular mechanism underlying this phenomenon remains mostly unknown, it has been suggested that it involves interactions between the natural product structure and constituents of the bacterial cell membrane, such as transmembrane proteins [37, 38].

Yousefzadi et al. [39] isolated *α*-pinene from the essential oil of *Salvia chloroleuca* and evaluated its antibacterial activity, demonstrating moderate and strong inhibitory activities against *S. aureus* and *E. coli*, respectively. However, no activity was found against *P. aeruginosa*, which can be explained due to differences in the structure of the cell membrane of Gram-positive and Gram-negative bacteria, in particular, the lipid bilayer [38, 40].

Da Silva et al. [17] evaluated the antimicrobial activity of pinenes, demonstrating that (-)-*α*-pinene and (-)-*β*-pinene had no significant antimicrobial activity at concentrations below 20 mg/mL, while the positive enantiomers showed inhibitory activities against methicillin-resistant *S. aureus* strains with MIC values ranging from 117 *μ*g/mL to 6,250 *μ*g/mL. Accordingly, the studies of Da Silva et al. [17] and Dhar et al. [41] found that (+)-*α*-pinene presented antibacterial activity against *S. aureus* strains. Moreover, De Sousa Eduardo et al. [42] and Freitas et al. [43] showed that *α*-pinene has promising effects against *S. aureus*, demonstrating a potential to be used in the combat of antibacterial resistance.

The results of the present work corroborate those presented by Da Silva et al. [17] who evaluated the combination of (+)-*α*-pinene and (+)-*β*-pinene with ciprofloxacin, showing synergistic activity against methicillin-resistant *S. aureus* (MRSA).

An antibiotic-potentiating effect was also obtained by Do Amaral et al. [44] who showed that the association of *α*-pinene with ceftazidime, amoxicillin, cefepime, cefoxitin, and amikacin resulted in enhanced antibiotic activity against *E. coli*.

This enhanced antibiotic effect may result from different mechanisms such as alteration in membrane permeability; inhibition of efflux pumps activity, or alteration in the expression of genes that codify proteins that mediate these mechanisms [45].

*S. aureus* can become resistant to antibiotics through genetic mutations that alter the target DNA gyrase or reduce outer membrane proteins, thus reducing drug accumulation [46, 47]. Martin et al. [48] reported a marked increase in resistance to trimethoprim-sulfamethoxazole in clinical isolates of *Staphylococcus aureus* and 7 genera of Enterobacteriaceae, including *E. coli*, from 1988-1995 at a hospital in California.

*E. coli* is naturally susceptible to almost all clinically relevant antimicrobial agents, in addition to being capable of accumulating resistance genes, mainly through horizontal gene transfer [49].

Studies performed by Breidenstein et al. [50] showed that *Pseudomonas aeruginosa* presents a high level of intrinsic resistance to most antibiotics, which can be explained by the restricted permeability of its outer membrane, in addition to the expression of efflux systems and antibiotic-inactivating enzymes such as *β*-lactamases.

Corroborating the results of this study, Ali et al. [51] evaluated *P. aeruginosa* isolates and found significant resistance to amikacin, while resistance to trimethoprim-sulfamethoxazole was described by Bayraktar et al. [52].

Barbosa [53] evaluated the essential oil of *Chamaemelum nobile*, which has *α*-pinene and *β*-pinene as major components. The oil strongly modulated the activity of amikacin activity against *P. aeruginosa* PA01, causing a 128-fold reduction in the MIC of this antibiotic, corroborating the results of this study.

Nitroimidazole prodrugs such as metronidazole are activated by the reduction of the nitro group, which occurs at low oxygen rates, since oxygen can inhibit metronidazole uptake. Thus, the effective use of nitroimidazoles is limited to anaerobic bacteria, protozoa, and microaerophiles [54–57], corroborating the resistance profile observed in this study.

It is known lipophilic substances like beta-caryophyllene can induce significant changes in the membrane structure, resulting in morpho-physiological damage, such as reduced membrane potential, cytochrome C/protein and radical loss, proton pump collapse, and ATP depletion, among other toxic effects [30, 58–63]. Accordingly, studies by Andrews et al. [63], Harrewijn et al. [64], and Singh et al. [65] state that the mechanism of action by *α*-pinene is associated with cell membrane damage.

Kovač et al. [66] evaluated the antibacterial activity of the negative enantiomer *α*-pinene at the concentration of 125 mg/L, showing that this compound increased the membrane permeability, in addition to inducing an intracellular accumulation of antibiotics due to the inhibition of antimicrobial efflux systems, providing further inhibition of antimicrobial resistance. A number of studies [63–66] have also demonstrated that pinene compounds have caused damage to the membrane, which may also explain its effects on antibiotic activity potentiation, as demonstrated in this research.

Badawy et al. [67] described the antimicrobial effects of various monoterpenes, among which thymol and *α*-terpineol had the most potent activity against *E. coli* and *S. aureus*. De Souza et al. [68] evidenced the efficacy of the association between carvone and penicillin against MRSA, as well as demonstrated the potentiating effects of eugenol and thymol associated with penicillin against beta-lactam-resistant *E. coli*. In corroboration, the work of De Souza et al. [68] found that d-limonene had a synergistic effect when associated with gentamicin against *S. aureus* and *E. coli* while the monoterpene geraniol enhanced the activity of kanamycin against the bacterial strain 358 of *S. aureus* [69].

Sill with regard to effects of monoterpenes against resistant *S. aureus* strains, Freitas et al. [43] also stated that *α*-pinene potentiated the effect of tetracycline against the *S. aureus* IS-58 strain, while studies with *E. coli* conducted by Pereira et al. [70] showed that the complex (+)-*β*-citronellol (*β*CT)/*β*-cyclodextrin (*β*-CD) in combination with gentamicin showed a synergistic effect against *E. coli*.

Research by Gachkar et al. [71] has attributed the antimicrobial activity of some essential oils to the presence borneol, which has been identified as a major constituent of the essential oils obtained from the flowers, leaves, and stem of *Rhynchanthus beesianus* [72], which presented significant antibacterial activity against *Bacillus subtilis*, *Enterococcus faecalis*, *S. aureus*, *Proteus vulgaris*, *P. aeruginosa*, and *E. coli*.

Studies on the antibacterial mechanism of action of terpenes [73–75] have indicated that the antimicrobial activities of thymol and carvacrol are associated with their ability to cause changes in membrane permeability. According to Breidenstein et al. [50], the restricted permeability of the outer membrane, as well as the presence of efflux systems, and the production of antibiotic-inactivating enzymes, such as *β*-lactamases, collaborate to the high level of antibiotic resistance observed in *Pseudomonas aeruginosa*, which could justify the lack of significant modulation of the antibiotic activity by the compounds evaluated in the present research. Finally, the present findings corroborate those obtained by Siddique et al. [76] who showed that borneol did not exhibit antibacterial activity against MDR clinical isolates of *S. aureus* and MRSA.

While specific mechanisms involved in the antimicrobial action of monoterpenes remain poorly characterized, studies by Sikkema et al. [61] and Sikkema et al. [11] have suggested that due to their lipophilic character, monoterpenes will preferentially divide from an aqueous phase into membrane structures, thus causing structural and functional damage, which has been used to explain the antimicrobial action of oils and their monoterpenoid components in most works. According to Trombetta et al. [77], the action of these compounds on the bacterial membrane leads to expansion, increased fluidity and permeability, disturbance of protein function, and inhibition of ion transport. Thus, the existence of certain epistatic interactions that result in variable responses in studies addressing different species and antibiotics cannot be ruled out.

Besides the antibacterial activity, research has demonstrated that borneol has analgesic, anti-inflammatory, antioxidant, healing, and antifungal activities [78, 79].

Yang et al. [79] reported that (+)-borneol (BNL1) and (-)-borneol (BNL2) can induce drug accumulation in cells due to its interference with P-glycoprotein (Pgp), an efflux protein that contributes to multidrug resistance to antibiotics and anticancer drugs, which could potentially explain the synergistic effects observed from the association between monoterpenes and antibiotics, as demonstrated in this work.

Of note, to date, no study evaluating the antibiotic-enhancing activity of (-)-borneol has been found in the literature, highlighting the pioneering aspect of the present research.

## 4. Conclusions

The results presented in this work suggest that (+)-*α*-pinene and (-)-borneol are promising compounds in the inhibition of antibiotic resistance, although further research is required to investigate both the safety and effectiveness of this combined treatment in the management of infections caused by *S. aureus*, *E. coli*, and *P. aeruginosa*.

The results of this work can contribute to the development of new antibacterial therapies using lower doses of monoterpenes and antibiotics, increasing the effectiveness and reducing the side effects resulting from antibiotic therapy.

## Figures and Tables

**Figure 1:** Antibiotic-modulating activity of (+)-*α*-pinene associated with antibiotics against *S. aureus*. TMP/SMX: trimethoprim/sulfamethoxazole. *p* < 0.0001 = ∗∗∗∗.

**Figure 2:** Antibiotic-modulating activity of (-)-borneol associated with antibiotics against *S. aureus*. TMP/SMX: trimethoprim/sulfamethoxazole. *p* < 0.0001 = ∗∗∗∗.

**Figure 3:** Antibiotic-modulating activity of (+)-*α*-pinene associated with antibiotics against *E. coli*. TMP/SMX: trimethoprim/sulfamethoxazole. *p* < 0.0001 = ∗∗∗∗.

**Figure 4:** Antibiotic-modulating activity of (-)-borneol associated with antibiotics against *E*. *coli*. TMP/SMX: trimethoprim/sulfamethoxazole. *p* < 0.0001 = ∗∗∗∗.

**Figure 5:** Antibiotic-modulating activity of (+)-*α*-pinene associated with antibiotics against *P. aeruginosa*. TMP/SMX: trimethoprim/sulfamethoxazole. *p* < 0.0001 = ∗∗∗∗.

**Figure 6:** Antibiotic-modulating activity of (-)-borneol associated with antibiotics against *P*. *aeruginosa*. TMP/SMX: trimethoprim/sulfamethoxazole. *p* < 0.0001 = ∗∗∗∗.

**Table 1:** Resistant profile of the strains.

Bacteria	Origin	Resistance profile
*Staphylococcus aureus* 10	Rectal swab	Amc, Amox, Amp, Asb, Azi, Ca, Cef, Cf, Cip, Cla, Clin, Eri, Lev, Mox, Oxa, Pen
*Pseudomonas aeruginosa* 24	Nasal discharge	Ami, Cip, Cpm, Ctz, Imi, Lev, Mer, Ptz
*Escherichia coli* 06	Urine culture	Asb, Ca, Cef, Cfo, Cmp, Cro

Subtitle: Amc: amoxicillin + clavulanic acid (20/10 *μ*g); Ami: amikacin (30 *μ*g); Amox: amoxicillin (20 *μ*g); Amp: ampicillin (10 *μ*g); Asb: ampicillin + sulbactam (10/10 *μ*g); Azi: azithromycin (15 *μ*g); Ca: cefadroxil (30 *μ*g); Cef: cephalexin (30 *μ*g); Cfo: cefoxitin (30 *μ*g); Cip: ciprofloxacin (5 *μ*g); Cla: clarithromycin (15 *μ*g); Clin: clindamycin (2 *μ*g); Cmp: cefepime (30 *μ*g); Cro: ceftriaxone (30 *μ*g); Ctz: ceftazidime (30 *μ*g); Eri: erythromycin (15 *μ*g); Imi: imipenem (10 *μ*g); Lev: levofloxacin (5 *μ*g); Mer: meropenem (10 *μ*g); Mox: moxifloxacin (5 *μ*g); Oxa: oxacillin (1 *μ*g); Pen: penicillin (30 *μ*g); Ptz: piperacillin (100 *μ*g) [40].

**Table 2:** Minimum inhibitory concentration of (+)-*α*-pinene and (-)-borneol.

Microorganisms	MIC	
	(+)-*α*-Pinene	(-)-Borneol
*E. coli*	512 *μ*g/mL	512 *μ*g/mL
*S. aureus*	≥1024 *μ*g/mL	≥1024 *μ*g/mL
*P. aeruginosa*	≥1024 *μ*g/mL	≥1024 *μ*g/mL

## Data Availability

The data used to support the findings of this study are available from the corresponding author upon request.
